The article "Development and validation of a prediction model for depression in adolescents with polycystic ovary syndrome: A study protocol" was published in 2022. Journal: Front Psychiatry.

# Development and validation of a prediction model for depression in adolescents with polycystic ovary syndrome: A study protocol

**DOI:** 10.3389/fpsyt.2022.984653

**Published:** 2022-09-06

**Authors:** Rui Ding, Heng Zhou, Xin Yan, Ying Liu, Yunmei Guo, Huiwen Tan, Xueting Wang, Yousha Wang, Lianhong Wang

**Affiliations:** ^1^Nursing Department, Affiliated Hospital of Zunyi Medical University, Zunyi, China; ^2^Nursing College, Zunyi Medical University, Zunyi, China; ^3^Reproductive Medicine Department, Affiliated Hospital of Zunyi Medical University, Zunyi, China

**Keywords:** polycystic ovary syndrome, adolescents, depression, prediction model, LASSO regression

## Abstract

**Introduction:**

The high prevalence and severity of depression in adolescents with polycystic ovary syndrome (PCOS) is a critical health threat that must be taken seriously. The identification of high-risk groups for depression in adolescents with PCOS is essential to preventing its development and improving its prognosis. At present, the routine screening of depression in adolescents with PCOS is mainly performed using scales, and there is no early identification method for high-risk groups of PCOS depression in adolescents. It is necessary to use a warning model to identify high-risk groups for depression with PCOS in adolescents.

**Methods and analysis:**

Model development and validation will be conducted using a retrospective study. The study will involve normal adolescent girls as the control group and adolescent PCOS patients as the experimental group. We will collect not only general factors such as individual susceptibility factors, biological factors, and psychosocial environmental factors of depression in adolescence, but will also examine the pathological factors, illness perception factors, diagnosis and treatment factors, and symptom-related factors of PCOS, as well as the outcome of depression. LASSO will be used to fit a multivariate warning model of depression risk. Data collected between January 2022 and August 2022 will be used to develop and validate the model internally, and data collected between September 2022 and December 2022 will be used for external validation. We will use the C-statistic to measure the model's discrimination, the calibration plot to measure the model's risk prediction ability for depression, and the nomogram to visualize the model.

**Discussion:**

The ability to calculate the absolute risk of depression outcomes in adolescents with PCOS would enable early and accurate predictions of depression risk among adolescents with PCOS, and provide the basis for the formulation of depression prevention and control strategies, which have important theoretical and practical implications.

The article "Development and validation of a prediction model for depression in adolescents with polycystic ovary syndrome: A study protocol" was published in 2022. Journal: Front Psychiatry.

**Trial registration number:**

[ChiCTR2100050123]; Pre-results.

## Introduction

Polycystic Ovary Syndrome (PCOS) is a female endocrine metabolic disease of unknown etiology, with a prevalence of 5.6 to 11.04% in adolescence (1) and 10.26% in the Chinese adolescent population (2). Symptoms of PCOS include abnormal menstruation, infertility, hyperandrogenismia, and polycystic ovarian changes (3). It has been controversial and challenging to diagnose PCOS during adolescence due to the overlap between regular pubertal physiological changes (irregular menstrual cycles, acne, and polycystic ovarian morphology on pelvic ultrasound) and adult PCOS diagnostic criteria. Consensus statements on adult and pediatric health have acknowledged these challenges (4–6). To be more specific, challenges include the risk of under-diagnosis, delayed and/or poor diagnosis experiences (7), and over-diagnosis, as well as the additional risk of the use of inconsistent non-evidence-based approaches to PCOS diagnosis and management (8). PCOS generally begins after the first menarche in adolescence and lasts through the reproductive years and perimenopause. Besides affecting reproductive health, PCOS increases the risk of diseases such as type 2 diabetes, cardiovascular disease and endometrial cancer (9), as well as the development of psychiatric disorders. Adolescent girls with PCOS are 2.4 times more likely to suffer from depression than normal girls of the same age, about 50–60% (10, 11). A depressive disorder can result in great psychological and physical distress in adolescents, leading to suicide in over half of them, and it can affect the health and psychosocial functioning of adults as well (12). Studies have shown that PCOS can also lead to infertility in the long run (13). Nevertheless, recent studies suggest that PCOS on its own is not necessarily a cause of infertility (14). It is possible that infertility can be exacerbated by emotional and psychiatric problems in PCOS patients due to illness and fear of future infertility (14). Thus, it is recommended that psychological, emotional, and other non-medical measures be optimized in order to treat infertility, as well as increasing the attention given to depression in individuals with PCOS. PCOS, however, has no identified etiology and no specific treatment. Life management is recommended by international evidence-based guidelines as the ideal treatment for PCOS (15), but patients with the disorder have poor life management skills (16). The guideline declares that patients with PCOS can participate in better life management by improving their psychological status (4). There is no doubt that depression is a significant health issue that must be addressed in the management of adolescents with PCOS.

The article "Development and validation of a prediction model for depression in adolescents with polycystic ovary syndrome: A study protocol" was published in 2022. Journal: Front Psychiatry.

Depression high-risk groups are individuals or subgroups who suffer from certain depressive symptoms but do not meet the diagnostic criteria for depression (17). They constitute a mental sub-health state between health and depression. Given the high prevalence of depression in adolescents with PCOS, warning of its onset risk and identification of high-risk groups is significant for preventing its development and improving its prognosis (18). There is currently no early detection approach for high-risk groups of depression in adolescents with PCOS, and most routine screening uses questionnaires. Hence, it's necessary to develop a warning model to identify adolescents with PCOS at high risk for depression.

The development of warning models often involves the incorporation of influencing factors. However, a variety of factors affect depression in adolescents, including: (i) biological factors, such as hormones and individual development during adolescence, which modifies neuroendocrine regulation and brain structure in diverse ways, contribute to adolescent depression. For instance, altering the activity of the hypothalamic-pituitary-adrenocortical (HPA) axis, affecting the release of neurotransmitters, altering the REM sleep latency, and so on, can all have an impact on the neurological structure and psychological state of the adolescent population, eventually leading to depression (19); (ii) individual susceptibility factors, such as genetic factors, with heredity influence approximately 40–50% of depressed people. Depressed people's first-degree relatives have a 10–13% chance of developing depression (20); (iii) psychosocial environmental factors, such as family environments, social development and social role changes, and negative behavior patterns, contribute to a sense of helplessness, which leads to negative attributions and ultimately to depression in the long run (21). PCOS may also be associated with several factors, such as insulin resistance and obesity, which may further aggravate the endocrine disorder during adolescence and increase the dysregulation of the HPA axis. Likewise, PCOS also leads to higher levels of androgen in the body, which is closely related to the risk factors of mental diseases (22), so there is speculation that pathological factors such as insulin resistance, obesity and high levels of androgen play a role in the occurrence of depression in PCOS (23). Hormonal drugs, like Ethinylestradiol cyproterone acetate tablets, are often used to treat PCOS. These drugs affect the cortical and subcortical areas of the brain that control emotions. These areas are immature and oversensitive in adolescents, which greatly increases the risk of depression (24). A lack of control over menstrual irregularities (11), as well as a lack of knowledge and information about the disease, which increases the psychological burden of the patients and may worsen depression (25). It can be seen that depression in PCOS is linked to the above-mentioned factors directly or indirectly. It's difficult to predict depression risk from one or more of these factors with any certainty because the number and magnitude of influencing factors are still inconclusive (Figure 1). Thus, developing a warning depression model for adolescents with PCOS through the interaction of complex influencing factors is a critical problem that requires immediate research, and there is no such report currently available.

The article "Development and validation of a prediction model for depression in adolescents with polycystic ovary syndrome: A study protocol" was published in 2022. Journal: Front Psychiatry.

**Figure 1:** Simulation map of risk factors for depression in adolescents with PCOS.

As previously noted, the occurrence of depression in adolescents with PCOS involves multiple dimensions and contains numerous independent variables. To minimize the bias caused by the absence of important independent variables, it's important to select as many variables as possible at the beginning of the warning model construction process. Traditional regression analysis methods using statistical software such as SPSS, Jamovi, etc., can quantitatively analyze the strength of a predictor based on the regression coefficient. However, conventional regression analysis methods cannot handle collinearity problems and produce high variance when there are numerous independent variables. Least Absolute Shrinkage and Selection Operator (LASSO) is a type of machine learning method introduced by Tibshiran in 1996 (26). On the one hand, LASSO can select features automatically. When there are numerous independent variables, LASSO can selectively integrate powerful explanatory factors into the model. On the other hand, LASSO can compress the coefficients of some minor or insignificant independent variables to zero and pick more relevant independent variables to prevent overfitting. As compared to traditional regression analysis methods, LASSO can process all independent variables simultaneously, which greatly increases the model's stability. LASSO has been gradually applied to the development of warning models in the medical area in recent years (27, 28), as it offers high stability, fast calculation speed, and ease of interpretation in building warning models. To date, LASSO has been applied to the construction of diagnostic prediction models, early risk identification of ischemic stroke, for example (27). LASSO has also been applied to the construction of prognostic prediction models, for instance, survival after ampullary adenocarcinoma resection (28). Additionally, a study based on LASSO used electronic primary care data to develop a predictive model of common mental disorders among adolescents and early adults (29). But the study noted that primary care data underestimated common mental disorders. Due to race and PCOS, the model cannot predict depression with PCOS in adolescents. Thus, we will explore the causes of depression in teenagers with PCOS and the influence of a variety of risk variables, as well as develop and test a depression risk prediction model for adolescents with PCOS. Not only will this model be able to identify high-risk groups for depression with PCOS in adolescence, but also for high-risk groups of depression in general adolescent girls.

The article "Development and validation of a prediction model for depression in adolescents with polycystic ovary syndrome: A study protocol" was published in 2022. Journal: Front Psychiatry.

## Objectives

The aims of the study are to: (i) Develop a depression prediction model for adolescents with PCOS to identify at-risk populations early; (ii) Validate the accuracy and validity of the model and to assess the clinical utility of the model.

## Methods and analysis

### Preparation

A multidisciplinary research team was established, consisting of obstetricians and gynecologists (*n* = 2), psychiatrists (*n* = 2), psychologists (*n* = 1), nursing specialists (*n* = 1), statisticians (*n* = 1) and research assistants (*n* = 2). Members of the research team have received uniform training in PCOS clinical practice and adolescents as well as extensive experience in their respective fields. Firstly, the team derived an understanding of depression among adolescent PCOS patients by retrieving evidence-based information and integrating clinical practices. Secondly, the research team reviewed the factors associated with depression in adolescents in the general population, and then the pathological factors of PCOS, the perception factors of PCOS, the diagnosis and treatment factors of PCOS, and the symptoms-related factors of PCOS, to summarize the risk factors for depression in adolescents with PCOS.

### Study design

We will use a retrospective cohort design for predictive model development and validation studies. It will follow expert guidance on model development and validation (30, 31), and reported per the Transparent Reporting of multivariable prediction model for Individual Prognosis or Diagnosis (TRIPOD) statement (32).

### Participants

The study will be conducted at the Affiliated Hospital of Zunyi Medical University in Zunyi, Guizhou Province. It is a 2,800-bed general hospital with over two million outpatient attendances per year. An average of 80–100 adolescent PCOS patients are seen at the gynecological clinic per month, providing the sample size required for this study.

The article "Development and validation of a prediction model for depression in adolescents with polycystic ovary syndrome: A study protocol" was published in 2022. Journal: Front Psychiatry.

### Patient recruitment

Adolescents with PCOS who attend the gynecology clinic of the Affiliated Hospital of Zunyi Medical University from January 2022 to August 2022 will be selected as the potential participants using a consecutive enrollment method. The final participants will be identified based on inclusion and exclusion criteria, and data are collected as both a training dataset and a validation dataset for the model construction. Data collected from September 2022 to December 2022 as an external validation cohort. Participants listed above will comprise the experimental group. Additionally, a control group will be recruited from the gynecology clinic among healthy, age-matched adolescent girls.

### Eligibility criteria

#### Inclusion criteria

1. Aged 10–19 years old (33).
2. According to “Chinese guidelines for diagnosis and treatment of polycystic ovary syndrome,” which was developed by the Endocrinology Group of the Chinese Medical Association Obstetrics and Gynecology Branch in 2018 (34), PCOS participants in the study must meet all three indicators in the Rotterdam diagnostic criteria at the same time (35), including: (i) oligomenorrhea persisting for at least 2 years after menarche, or amenorrhea; (ii) clinical manifestations of hyperandrogenism or hyperandrogenemia; (iii) the diagnosis of PCO on ultra sound includes increased ovarian size (>10 cm^3^).
3. Able to self-report (verbally understandable and articulate).
4. Participants and their families volunteer to participate in the study.

#### Exclusion criteria

1. Participants with cognitive impairment and major mental illness (36)(schizophrenia, schizoaffective disorder, bipolar disorder, etc.) (37).
2. Participants with serious comorbidity(Other diseases that seriously affect the patient's normal life, such as acute myocardial infarction, systemic lupus erythematosus complicated by severe renal dysfunction, etc.).
3. Other conditions that lead to elevated androgen levels (congenital adrenal cortical hyperplasia, Cushing syndrome, androgen-secreting tumors, etc.) and cause ovulation disorders (hyperprolactinemia, premature ovarian failure, functional hypothalamic amenorrhea, thyroid dysfunction, etc.).

### Determinations and variables

After discussion and conclusion, the research team obtained indicators of independent and dependent variables affecting depression in PCOS adolescents, as follows.

#### Dependent variables

Depression will be measured by the Chinese version of the Children's Depression Scale(CDI) (38). The scale is comprised of 27 items, each of which offers three possible replies based on the respondent's actual mood during the previous 2 weeks. The project consists of five dimensions: anhedonia, poor efficacy, low self-esteem, negative emotions, and interpersonal problems. The intensity of each item determined whether it was rated zero, one, or two, and the negative word statement was scored in reverse. A score of 19 indicated the presence of depressive symptoms. It has been reported that the Chinese version of the CDI scale has been applied to children and adolescents ranging from 7 to 18 years of age in China (38–40). CDI has the advantage of having the lowest reading level of all depression measurement tools (only the first grade level). The Chinese version of the CDI scale has a good level of reliability and validity, as well as a high clinical diagnostic value for depression, and can be used to measure depression in children and adolescents in China. Utilize the total score to reflect the severity of depressive symptoms or diagnostic threshold due to its operability and clinical applicability.

The article "Development and validation of a prediction model for depression in adolescents with polycystic ovary syndrome: A study protocol" was published in 2022. Journal: Front Psychiatry.

We will use the Kiddie-Schedule for Affective Disorders and Schizophrenia-Epidemiological version (K-SADS-E) to confirm the diagnosis of depression and exclude possible comorbidities. The validated Mandarin version will be used in this study (41). It is a semi-structured diagnostic interview questionnaire designed to assess the current and past mental health status of children and adolescents aged 6-18 in accordance with the diagnostic criteria of the Diagnostic and Statistical Manual of Mental Disorders, 5th edition (DSM-5). In this study, two psychiatrists trained in K-SADS-E interview harmonization will conduct interviews to diagnose depression and exclude possible comorbidities. It will take approximately 1–1.5 h for each participant and their parents to complete the interview. It has been demonstrated that K-SADS-E has good psychometric properties (41). The diagnoses of K-SADS-E demonstrated good convergent and divergent validity with most corresponding clinical questionnaires.

#### Independent variables

The predictors for building the model are shown in Table 1.

**Table 1:** Model-building predictors: definition/measuring tools, variable type and units/categories.

**Candidate predictor**	**Definition/Measuring tools**	**Variable type**	**Units/categories**
**Individual susceptibility factors**			
Age	Adolescent's age	Continuous & Categorical	Years (age classified into approximately three to four categories)
Nationality	Adolescent's nationality	Binary	0 “the Han nationality” 1 “minority nationality”
Body mass index(BMI)	Body mass divided by the square of the body height	Continuous	kg/m^2^
Waist-to-hip ratio (WHR)	WHR is found by dividing circumference of the waist by the circumference of the hips	Continuous	
Living residence	Current residence of adolescents	Binary	0 “City” 1 “Countryside”
Education level	Current educational level of adolescents	Categorical	Education level classified into approximately five categories
Single parent family	Adolescents live with only one parent	Binary	0 “No” 1 “Yes”
Family history of mental illness	Mental illness within three generations in the paternal, maternal, direct and collateral lines in adolescents	Binary	0 “No” 1 “Yes”
Duration of illness	Time since first diagnosis of PCOS	Categorical	Duration of illness classified into approximately five to six categories
Personality	Eysenck Personality Questionnaire-Junior (42)	Continuous	
Emotional regulation skills	Emotion Regulation Scale (43)	Continuous	
**Diagnosis and treatment factors**			
Medication use	Adolescents with PCOS taking some medications, such as metformin, oral contraceptives and so on. If yes, please specify the medicine	Binary & Categorical	0 “No” 1 “Yes” (medications classified into approximately four to five categories)
Duration of medicine use	Duration of medicine use since first diagnosis of PCOS	Categorical	Duration of medicine use classified into approximately five to six categories
**Biological factors**			
Sleep	Athens Insomnia Scale (44)	Continuous	
**Psychosocial environmental factors**			
Interpersonal sensitivity	Symptom Checklist-90 (45)	Continuous	
Social support	Medical Outcomes Study Social Support Survey (46)	Continuous	
**Clinical symptoms**			
Hirsutism	Ferriman-Gallwey Rating Scale (47)	Continuous	
Acne	Rosenfield Scale (48)	Continuous	
Body image	The Nagetive Physical Self Scale (49)	Continuous	
**Illness perception factors**			
Illness perception	The Brief Illness Perception Questionnaire (50)	Continuous	
**Laboratory investigations**			
Sex hormone-binding globulin	Electro chemiluminescent immunoassay(ECLIA)	Continuous	nmol/L
Free testosterone index		Continuous	
Estradiol		Continuous	pmol/L
Follicle stimulating hormone		Continuous	mIU/mL
Luteinizing hormone		Continuous	mIU/mL
Progesterone		Continuous	nmol/L
Prolactin		Continuous	mIU/L
Total testosterone		Continuous	nmol/L
Dehydroepiandrosterone sulphate		Continuous	μmol/L
Third-generation thyrotropin		Continuous	μIU/mL
Insulin		Continuous	μIU/mL

The article "Development and validation of a prediction model for depression in adolescents with polycystic ovary syndrome: A study protocol" was published in 2022. Journal: Front Psychiatry.

### Data collection

Two uniformly trained researchers will identified participants based on inclusion and exclusion criteria. Firstly, a researcher will guide participants and their parents to a quiet outpatient room that is conducive to dialogue and data collection. Another researcher will explain the purpose, significance, and implementation of the study to participants and their parents in a one-on-one format, assuring them that their privacy would be protected. With the consent of participants and their parents, researchers will sign informed consent forms with them. Afterwards, psychiatrists within the study team will conduct semi-structured interviews with participants and their parents, focusing on the diagnosis of depression and excluding possible comorbidities. The researchers will distribute the QR code of the scale that was included in the questionnaire platform in advance to participants who are eligible, and the participants will scan the QR code on WeChat to fill out the form online. Finally, the researchers will give the participants health education and prescription advice, as well as recording laboratory indicators including sex hormones and insulin. The total planned time for this process will be around 2 h. The data will be extracted *via* a questionnaire platform and collated into Excel format, with the two researchers collecting the information independently and negotiating any disagreements.

### Quality control

1. The screening process will strictly adhere to the inclusion and exclusion criteria.
2. Prior to conducting formal research, researchers will receive standardized training.
3. Before the survey, researchers will explain the contents and precautions of the questionnaire to participants and their families. To ensure participants understand items, researchers will use uniform language to explain them, while avoiding leading words.
4. The questionnaire must be completed without omissions to ensure completeness of content and efficient recall.
5. Two researchers check and correct any discrepancies with the original data to ensure accuracy.

### Sample size and calculation

In the case of a binary outcome, an approximate 95% confidence interval for the total outcome proportion (ϕ) is


$$\begin{array}{l} \hat{\phi }\pm 1.96\sqrt{\frac{\hat{\phi }\left(1-\hat{\phi }\right)}{n}}, \end{array}$$

Therefore, the absolute margin of error (δ) is $1.96\sqrt{\frac{\hat{\phi }\left(1-\hat{\phi }\right)}{n}}$

For this reason, in order to get an accurate estimate of the overall outcome probability in the target population, based on the expected outcome proportion ($\hat{\phi }$) and the desired margin of error, the required sample size is calculated as: $n={\left(\frac{1.96}{\delta }\right)}^{2}\hat{\phi }\left(1-\hat{\phi }\right)$.

In general, we advise aiming for a margin of error of <0.05. Then assuming an anticipated outcome proportion in the study population of 0.4, then a minimum of 369 participants is needed to aim for an estimation error of no more than 0.05 around the actual value of 0.4 (51).

The article "Development and validation of a prediction model for depression in adolescents with polycystic ovary syndrome: A study protocol" was published in 2022. Journal: Front Psychiatry.

The study will include all adolescents with PCOS who attend the gynecology clinic of the Affiliated Hospital of Zunyi Medical University between January 2022 and December 2022, with an estimated sample size of 800. This study will recruit 400 healthy adolescent girls as the control group.

### Statistical analysis methods

The data obtained will be analyzed using SPSS Statistics version 18 (IBM Corp) software and evaluated using comparative and descriptive statistics. Student *t*-test will be used for normally distributed parametric data, while Mann-Whitney U-test will be used for non-normally distributed data. The χ^2^ test and Fisher exact test will be used to evaluate categorical data. A correlation between data will be evaluated using Pearson correlation coefficients for parametric data and Spearman correlation coefficients for non-parametric data. Descriptive statistics will be presented as median (range), mean ± SD, or number/frequency (percentage). Statistics will be considered significant when the *P*-value < 0.05.

#### Handling of predictors

The collected data will first be preprocessed, including data cleansing, outlier processing, and data transformation. Data cleaning is the process of deleting redundant information and correcting information with obvious errors. Based on the data situation, we will choose between deletion, imputation, or substitution for outlier processing. The data will be transformed in the following ways: continuous variables will be kept in the model as continuous variables if they are linear or will be combined with similar segments if they are non-linear (treated as binary categories or ordered categories); ordered multicategorical variables will be treated as rank variables or dummy variables as appropriate, and when not linearly related to the outcome, optimal scale regression will be used to explore effect inflection points; unordered multicategorical variables need to be split into multiple binary variables (Figure 2).

**Figure 2:** Simulation diagram for developing and validating a LASSO-based model to predict depression in adolescents with PCOS.

Preprocessed data will be assigned variable values according to various variable types and a data set in CSV format will then be generated.

#### Model-building procedures (including predictor selection)

After the data set is imported into the R software, it will be divided into 80% training data and 20% validation data. The training data will be used to build the warning model, and the validation data will be used for internal validation.

To begin with, we will use R software to read the features of the dataset. After that, we will load the two R packages “corrplot” and “glmnet.” By using the cor() function, we will create a correlation object “corrlate” and visualize the correlation coefficient. The predictors and outcome variables in the training and validation sets will be encoded into matrices, the predictors will be stored in X vectors, and the outcome variables in Y vectors. A LASSO regression will be performed when alpha is set to one. The program will then be run. When the parameter lambda is greater, the estimated parameters will also be compressed to a smaller degree. As lambda reaches a certain value, some variables that are not important to the model will be compressed to zero, indicating that these variables will be eliminated. Thus, the lambda corresponding to the optimal result, the influencing factors of preliminary screening, and the regression coefficient will be obtained.

The article "Development and validation of a prediction model for depression in adolescents with polycystic ovary syndrome: A study protocol" was published in 2022. Journal: Front Psychiatry.

#### Internal validation and assessment of model performance

Internal validation will be conducted using the 20% validation set samples and will utilize a cross-validation method based on 10 folds. Then, the result of LASSO cross-validation will be obtained, and the lambda when it is one standard error away from the mean square error will be considered optimal (at this time, the mean square error is small, and the number of independent variables is also small). For that lambda case, we will examine the regression coefficients and exclude variables with a regression coefficient of zero. Those variables with regression coefficients other than zero are selected, thereby identifying the influencing factors that are significantly associated with depression in PCOS adolescents. After screening the variables, a multivariate linear model will be constructed.

The prediction accuracy of the model will be reflected by discrimination and calibration. In this study, the C-statistic is used to measure discrimination, followed by a calibration plot to measure the accuracy of the absolute risk predictions of the warning model. An evaluation of the fit will be performed by drawing a scatter plot.

#### External validation

External validation will be conducted using temporal validation with data collected from September 2022 to December 2022, to ensure model portability and generalizability. This means that model risk scores will be calculated rigorously and the model will be refitted in the validation cohort.

After the model is defined, we will consider the nomogram as the final presentation form in order to facilitate clinical application of the model and assist medical personnel in identifying high-risk groups of depression in adolescents with PCOS.

All statistical analysis will be performed using R software (Windows version 4.1.2).

The article "Development and validation of a prediction model for depression in adolescents with polycystic ovary syndrome: A study protocol" was published in 2022. Journal: Front Psychiatry.

### Data storage and management

Data will be entered and stored through a third-party electronic platform, and all documents and data will be password-protected on a network within the platform, accessible only to researchers. Data will be exported in Excel format for further analysis when processed.

## Discussion

This research protocol aims to construct and validate a warning model for depression in adolescents with PCOS. It will answer three questions: what factors influence depression risk in adolescents with PCOS; what role do various types of depression risk factors play in the development of depression in adolescents with PCOS; and how interpretable and accurate is the LASSO-based warning system.

There are many factors associated with depression in adolescents with PCOS. For the first time, a depression warning model will be constructed that takes into account not only general factors like individual susceptibility factors, biological factors, and psychosocial environmental factors of depression in adolescence, but also the pathological factors, illness perception factors, diagnosis and treatment factors, and symptom-related factors of PCOS. This study will precisely and early identify depression at-risk groups for PCOS in adolescence by including the influencing factors of several dimensions of depression into the model and leveraging LASSO's ability to automatically screen variables and boost model interpretability.

So far, it has been difficult to identify adolescents at high-risk of depression, which has a severe impact on adolescent mental health. In this study, the research population consists of adolescents with PCOS, who have a significantly greater prevalence of depression and more complicated impacts than general adolescent girls, an important representative sample. Through this study, we hope to remove the bottleneck of identifying adolescents at risk of depression. The success of this study can not only identify the high-risk groups of depression in adolescents with PCOS, but also demonstrate the risk factors and key links associated with depression in adolescents with PCOS. At the same time, it can be extended and applied to the management of high-risk groups of depression throughout adolescent girls, thereby contributing to reducing the prevalence of depression in adolescent girls and implementing comprehensive and effective prevention measures.

The study is a retrospective cohort study, and the questionnaire will be partially completed by patients' recollection of recent events, which may be subject to a degree of recall bias. In prospective cohort studies, depression outcomes and factors contributing to depression can be longitudinally tracked over a period of time of high-risk groups with PCOS in adolescence, which can help to make models more robust and representative. Data for this study will be collected at one hospital, so it will be a single-center study. It is proposed that future studies should collect data from multiple hospitals simultaneously to increase sample size and persuasiveness. In this study, participants will be selected in accordance with the diagnostic criteria prescribed in the “Chinese guidelines for diagnosis and treatment of polycystic ovary syndrome.” Due to the inconsistency in diagnostic criteria among different ethnic groups, the generalizability of this study is limited to some degree. It is recommended that metformin and oral contraceptives be used to treat PCOS in adolescence, in accordance with international evidence-based guidelines (4). It has been reported, that oral contraceptives may increase participants' risk of depression (24), whereas metformin can help to alleviate depression (52). Hence, confounding effects may occur if participants take metformin and oral contraceptives concurrently. As part of our investigation, we will assess the medication status of the participants. However, we will not be able to eliminate the possibility that there may be a confounding effect. The model was externally validated using temporal validation, as the data source is the same as the model development cohort, which may be less transferable and generalizable than geographical validation (which validates the model against data from other centers or even other countries).

The article "Development and validation of a prediction model for depression in adolescents with polycystic ovary syndrome: A study protocol" was published in 2022. Journal: Front Psychiatry.

## Ethics statement

The studies involving human participants were reviewed and approved by the Ethics Committee of ZunyiMedical University: Zunhe Lun Review [2021] 1-093. Written informed consent to participate in this study will be provided by the participant's legal guardian/next of kin. Written informed consent will be obtained from the individuals and minor's legal guardian/next of kin, for the publication of any potentially identifiable images or data included in this article.

## Author contributions

RD was involved in writing the protocol, editing the manuscript, setting up the trial, and acquisition of data. HZ, XY, YG, YL, HT, XW, and YW participated in the design of the trial, analysis, and interpretation of the data. LW carried out the conception, design, and final approval of the version to be published and agreed to be accountable for all aspects of the work by ensuring that any questions regarding the accuracy or integrity of any part of the work are appropriately investigated and resolved. All authors contributed to the article and approved the submitted version.

The article "Development and validation of a prediction model for depression in adolescents with polycystic ovary syndrome: A study protocol" was published in 2022. Journal: Front Psychiatry.

## Funding

The work is supported by Zunyi Science and Technology Planning Project [Zun Shi Ke He HZ Zi (2021) No. 21]. The Science and Technology Department of Guizhou Province, China [Grant No. Qian Ke He (2017) 5733-077]. The Health Commission of Guizhou Province, China (Grant No. Gzwjkj2019-1-018).

## Conflict of interest

The authors declare that the research was conducted in the absence of any commercial or financial relationships that could be construed as a potential conflict of interest.

## Publisher's note

All claims expressed in this article are solely those of the authors and do not necessarily represent those of their affiliated organizations, or those of the publisher, the editors and the reviewers. Any product that may be evaluated in this article, or claim that may be made by its manufacturer, is not guaranteed or endorsed by the publisher.
